The article "Osthole Induces Apoptosis and Inhibits Proliferation, Invasion, and Migration of Human Cervical Carcinoma HeLa Cells" was published in 2021. Journal: Evid Based Complement Alternat Med.

# Osthole Induces Apoptosis and Inhibits Proliferation, Invasion, and Migration of Human Cervical Carcinoma HeLa Cells

**DOI:** 10.1155/2021/8885093

**Published:** 2021-09-09

**Authors:** Sugai Yin, Hejuan Liu, Jing Wang, Shuying Feng, Yulong Chen, Yiwan Shang, Xiuhong Su, Fuchun Si

**Affiliations:** Henan University of Chinese Medicine, No. 156 Jinshui East Road, Zhengzhou, Henan 450046, China

## Abstract

**Purpose:**

To study the effect of osthole extract on proliferation, migration, invasion, and apoptosis of human cervical carcinoma HeLa cells and investigate its underlying mechanism.

**Methods:**

HeLa cells were exposed to osthole at various concentrations. Cell viability, migration, and invasion were detected by MTT assay, scratch wound-healing assay, and invasion assay, respectively. The proportion of cells undergoing apoptosis was analyzed by flow cytometry. Western blot and RT-qPCR were performed to determine changes in the expression of key factors in the Wnt/*β*-catenin signaling pathway.

**Results:**

The osthole extract effectively inhibited the proliferation, migration, and invasion potential of HeLa cells in a dose-dependent manner. The rate of apoptosis induction in HeLa cells treated with the osthole extract for 48 h was significantly higher than that of the untreated controls. Outcomes of the western blotting analysis and RT-qPCR showed that the expression of *β*-catenin, c-Myc, cyclin D1, survivin, and MMP-9 was significantly inhibited.

**Conclusion:**

Osthole could significantly inhibit the malignant behavior of HeLa cells and induce cellular apoptosis. Inactivation of the Wnt/*β*-catenin signaling pathway by osthole may be a mechanism to control cancer metastasis.

## 1. Introduction

Cervical cancer is one of the most common female genital malignancies worldwide that pose a serious threat to the life and health of women aged 20 to 39 years [1, 2]. Cancer Statistics (2016) showed that about 520,000 new cases of cervical cancer were diagnosed annually, and nearly 70,000 people died from this fatal disease [3]. Currently, combined radiotherapy and chemotherapy remains the mainstay of treatment for cervical cancer and has demonstrated significant progress in cancer control. However, clinical complications of anticancer therapies or their severe side effects cannot be ignored.

In the past decades, Chinese medicine therapy has shown remarkable potential as an alternative for cervical cancer treatment or as auxiliary reagents that support cancer treatment owing to their high efficiency and low toxicity [4]. An increasing number of natural antineoplastic agents were employed in the preclinical and clinical assessments. For example, *in vitro* and *in vivo* studies on human cervical cancer suggested that Guizhi-Fuling-decoction, a traditional Chinese medical formulation, inhibited cervical cancer growth and metastasis [5]. *Fructus Cnidium* is a commonly used Chinese medicine in the clinic and is characteristically spicy, bitter, and warm. As recorded in “Shen Nong Ben Cao Jing,” it can warm the kidneys and activate Yang action, dry dampness, and insecticidal effect. Currently, it is widely applied in the treatment of morbid leukorrhea in women. Accumulating studies demonstrated that osthole, the main chemical constituent from *Fructus Cnidium*, presented a strong inhibitory effect on the growth of various tumor cells, such as lung cancer, colon cancer, breast cancer, and liver cancer [6–8]. It has been reported that osthole can induce cancer cell apoptosis and cell cycle arrest and inhibit tumor angiogenesis by manipulating some oncogenic signaling cascades, such as NFKB and PI3K signaling pathways [9, 10]. However, the pharmacological effects and mechanisms of osthole on cervical cancer were not very clear. This study aimed to assess the inhibitory effect of osthole on cervical cancer cells and explore its underlying mechanism in order to provide experimental evidence for clinical treatment of cervical cancer.

## 2. Materials and Methods

### 2.1. Materials and Reagents

Osthole (formula: C_15_H_16_O_3_, molecular weight: 244.29, specification: 20 mg, batch number: MUST–1708051, purity >98%) was procured from Chengdu Manst Biotechnology Co., Ltd. A stock solution of 10 mg osthole dissolved in 1 ml DMSO was prepared for the next dilution. Other reagents and kits used in the study included pancreatin (Suo Lai Bao company), RPMI1640 medium (Suo Lai Bao company), fetal bovine serum (Gibco company), and Annexin V-FITC/PI Apoptosis Detection Kit (KK Biotech, apoptosis kit: KGA172).

### 2.2. Cell Culture

The human cervical carcinoma HeLa cell line was obtained from the molecular biology testing center of the Henan University of Chinese Medicine. These cells were cultured in RPMI 1640 supplemented with 10% fetal bovine serum (FBS) and were maintained at 37°C in a humidified atmosphere with 5% CO_2_.

### 2.3. Cell Proliferation Assays

HeLa cells (1 × 10^4^) were plated in a 96-well plate. After culturing for 24 h, the old culture medium was discarded and it was substituted with a fresh medium containing different doses of osthole (from 50 and 100 to 200 *µ*g/mL) in 100 *µ*L. After treatment for 24 h, 48 h, and 72 h, respectively, 15 *µ*L of MTT dye solution (5 mg/mL) was added to each well and cell samples were incubated at 37°C for 4 h. The cultured product was dissolved by adding 150 *µ*L of DMSO to each well, and the plates were then read at 570/630 nm. The HeLa cells in the medium containing equal DMSO served as negative controls.

### 2.4. Scratch Wound-Healing Assay

HeLa cells were grown in a 24-well tissue culture plate at the density of 2 × 10^5^ cells/well overnight and then allowed to form a monolayer with ∼70–80% confluence. Straight lines were drawn across the surface of the well, and the equal gaps on the monolayer were marked. Cells were replenished with a fresh medium containing different concentrations (0, 50, 100, and 200 *µ*g/mL) of osthole followed by 48 h of subsequent culture. Scratch wounds were visualized on a microscope, and the gap distance was quantified with ImageJ software.

### 2.5. Cell Invasion Assay

To measure the cell invasive capacity, Millicell Cell Culture inserts were precoated with Matrigel. 2 × 10^4^ cells of different treated groups were maintained in the upper Transwell compartments, and the lower compartments were filled with the fresh medium. The cells were incubated at 37°C and 5% CO_2_ for 2.5 h and allowed to invade the other side of the insert filter. Next, the insert filter was fixed with 5% glutaraldehyde for 10 min and stained with 1% crystal violet in 1% ethanol for 15 min. The cells that transgressed through the membrane were regarded to possess invasive capacity and were counted under a microscope at ×100 magnification.

### 2.6. Detection of Apoptosis

Flow cytometry was used to detect HeLa apoptosis after treatment with different concentrations of osthole (0, 50, 100, and 200 *µ*g/mL). 1 × 10^5^ cells/well were seeded in a 6-well plate. The control group was cultured in a medium containing an equal concentration of DMSO. After 48 h of culturing, cells were digested using trypsin without EDTA. The treated cells were collected and washed twice with PBS, 1 × 10^5^ cells were counted in the flow tube and suspended in binding buffer and Annexin V-FITC for 10 min in the dark, and after that, propidium iodide (PI) was added to each sample for 5 min in the dark. Within an hour, apoptotic cells were measured using a FACS Calibur Flow Cytometer apparatus according to the manufacturer's instructions. At least three independent experiments were performed for each assay.

### 2.7. Western Blot

Cell lysates were prepared in 1x SDS sample buffer, and the protein content was calculated via the BCA protein content test kit as instructed. The sample protein (20 *µ*g) was loaded to slots of the gel in the electrophoresis chamber and resolved on 8% SDS-PAGE. Next, the proteins were transferred to a nitrocellulose membrane in a tank blot device at 15 V per gel and 4°C overnight. The membrane was incubated with 10 mL blocking solution for 1 h and then probed with 5 *µ*L primary antibodies for 3 h and horseradish peroxidase-conjugated goat anti-mouse for 1 h. Finally, the blots were developed with a chemiluminescence substrate solution ECL and exposed to X-ray films. *β*-Actin served as the reference gene to normalize gene expression.

### 2.8. Reverse Transcription-Quantitative PCR (RT-qPCR)

Total RNA was isolated from cells with the TRIzol reagent and reverse transcribed to T-cDNA using oligo-dT primers. T-cDNAs were amplified and quantified by qPCR with Mx3005P (Stratagene, USA), and expressions of *β*-catenin, c-Myc, cyclin D1, survivin, and MMP-9 gene were assessed. *β*-Actin served as the reference gene to normalize gene expression.

### 2.9. Statistical Analysis

Statistical analyses were conducted using Prism 8. Multiple group differences were analyzed by one-way and two-way ANOVA (for related genes expression). If statistical differences existed, the *t*-test was performed for comparison of two groups. Differences were considered statistically significant at *P* < 0.05.

## 3. Results

### 3.1. Osthole Inhibited Cell Proliferation of HeLa Cells

To determine the effect of osthole on human cervical carcinoma HeLa cells, we first investigated the proliferation and viability of HeLa cells by MTT assay after treatment with different doses of osthole for 24 h, 48 h, and 72 h. As illustrated in Figure 1, the cell viability of HeLa cells was significantly inhibited by osthole in a dose- and time-dependent manner (*P* < 0.01). These results demonstrated that osthole exhibited a pronounced antiproliferative effect on the viability of HeLa cells.

### 3.2. Osthole Induces Morphological Alteration and Apoptosis of HeLa Cells

Considering the cytotoxic effect of osthole, the cellular apoptosis was observed. As presented in Figure 2(a), treatment with 0 *μ*g/mL osthole just displayed 10.57 ± 0.52% apoptotic rate, whereas 50 *μ*g/mL osthole treatment increased the apoptotic rate to 30.12 ± 0.12%. The apoptotic cell proportions were considerably enhanced with the increase in concentration of osthole (Figure 2(b)). The expression of cleaved-caspase-3 was also reduced along with the increasing concentration of osthole (Figure 2(c)).

### 3.3. Osthole Inhibited the Migration and Invasion of HeLa Cells

Next, we performed the scratch wound-healing assay and Transwell invasion assay to monitor the effect of osthole on the migration and invasion of HeLa cells. The wound-healing assay revealed that HeLa cells exposed to osthole exhibited significant dose-dependent suppression in wound closure due to the impairment of the cell (Figures 3(a) and 3(b)). The invasive potential of osthole-treated HeLa cells was observed to be dose-dependently subdued as compared with the control group in the Transwell invasion assay (Figures 3(c) and 3(d)).

### 3.4. Osthole Inactivated the Wnt/*β*-Catenin Signaling Pathway

Wnt/*β*-catenin is reportedly the functionally dynamic and pleiotropic signaling pathway in various cellular behaviors, such as proliferation, apoptosis, and migration. Inactivating the Wnt/*β*-catenin signaling pathway has been established to be associated with the malignant nature of cancers, including human cervical carcinoma. *β*-Catenin, c-Myc, cyclin D1, survivin, and MMP-9 are regarded as the key manipulators in this signaling cascade [11–13]. Hence, we examined their expression after treatment with osthole and unveiled that the expression of *β*-catenin was considerably inhibited upon treatment in a dose-dependent way (Figure 4(a)). The simultaneous suppression in the expression of c-Myc, CCND1, CTNNB1, survivin, and MMP-9 was also observed by RT-qPCR and western blot (Figures 4(b) and 4(c)). The above outcomes suggest that osthole inhibited the Wnt/*β*-catenin signaling pathway.

## 4. Discussion

Previous investigations on osthole also reported its antitumor effects and inhibitory action on malignant behavior of cervical cancer cells [14, 15]. However, the mechanism is not fully understood. In this study, we evaluated the antitumor effects of osthole on HeLa cells and investigated the potential mechanism. The data showed that osthole could suppress the proliferation of HeLa cells, both dose- and time-dependently. Additionally, the inhibitory effect was also observed in the migration and invasion potential of HeLa cells.

Apart from excessive proliferation, tumor cells reportedly can escape normal apoptosis and resist cell death, finally contributing to tumorigenesis and cancer pathogenesis [16, 17]. Over the last two decades, researchers focused on the anticancer activity of osthole in different cancers. For example, osthole inactivates PI3K/AKT signaling pathway and represses the malignant phenotypes of gastric cancer cells [18]. Its anticancer ability was also described in pancreatic cancer [15], gallbladder cancer [19], and ovarian cancer [20]. In cervical cancer, Su et al. demonstrated that osthole showed increase in the inhibition of cisplatin on NRF2 expression, thereby eliminating drug resistance of tumor cells [21]. Che et al. also demonstrated that osthole blunted NF-*κ*B signaling and increased the irradiation sensitivity of tumor cells [9]. In line with the previous investigation in other cancer cells, we also found that osthole can significantly trigger apoptosis and inhibit the proliferation and migration of HeLa cells in a dose-dependent manner [22–24].

The Wnt/*β*-catenin pathway has been reported to play an important role in the occurrence and development of cervical carcinoma [11, 13]. Inactivation of *β*-catenin in cervical carcinoma cells can significantly attenuate the malignant cellular phenotypes, including cell proliferation, apoptosis, migration, and aggressiveness. It is also reported that activation of the Wnt/*β*-catenin pathway can promote the epithelial-to-mesenchymal transition of cervical carcinoma cells [25]. Hence, Wnt/*β*-catenin signaling cascade is regarded as a critical point of targeted therapy in cervical carcinoma patients. Expectedly, we found that *β*-catenin expression was significantly inhibited in HeLa cells upon treatment with osthole at various concentrations. Meanwhile, we measured several critical downstream factors of the Wnt signaling pathway, including c-Myc, CCND1, survivin, and MMP-9, and found that their expressions were also reduced. All results demonstrated that osthole might govern the malignant behaviors of cervical carcinoma cells by attenuating the Wnt/*β*-catenin pathway. Of note, osthole reportedly blunted NF-*κ*B signaling to repress the cervical carcinoma. Therefore, the anticancer properties of osthole might be a complex scenario. In the next work, we will focus on it.

In conclusion, our findings indicate that osthole mediates its antitumor effect on cervical carcinoma HeLa cells by inactivating the Wnt/*β*-catenin pathway. Our study may shed novel light on the therapy of cervical carcinoma.

## Figures and Tables

**Figure 1:** Cytotoxicity of osthole in HeLa cells. The suppressive effect of HeLa cell proliferation by treatment with osthole (50, 100, and 200 *µ*g/mL) evaluated by MMT assay (24, 48, and 72 h). Data were expressed as mean ± SEM (*n* = 5).

**Figure 2:** Cell apoptosis of HeLa cells evaluated by flow cytometry. (a, b) HeLa cells were subjected to osthole (0, 25, 50, and 100 *µ*g/mL) and maintained for 48 h. ^*∗∗∗∗*^*P* < 0.0001. (c) Western blot analysis of caspase-3 expression in HeLa cells subjected to osthole (0, 25, 50, and 100 *µ*g/mL) and maintained for 48 h.

**Figure 3:** Effect of osthole on migration and aggressiveness of the HeLa cell. (a, b) Wound-healing assays were executed on HeLa cells, and the cell migration was evaluated after treatment with 0, 25, 50, and 100 *µ*g/mL of osthole for 24 h. Osthole attenuated cell migration and impaired the recovery of the HeLa monolayer. (c, d) Transwell invasion assays were carried out to test the cell invasion after treatment with 0, 25, 50, and 100 *µ*g/mL of osthole for 24 h and showed that osthole significantly inhibited cell invasion. ^*∗∗∗∗*^*P* < 0.001.

**Figure 4:** Osthole considerably suppressed the expression of c-myc, CCND1, survivin, MMP-9, and *β*-catenin. (a, b) *β*-Catenin protein expression in HeLa cells treated with osthole as detected by western blot. (c) RT-qPCR-based quantification of the mRNA expression of c-myc, CCND1, survivin, and MMP-9. (d) Western blot assessing the c-myc and CCND1 expression.

## Data Availability

The data used during the current study are available from the corresponding author on reasonable request.
